RETRACTED

# Neuromuscular electrical stimulation in critically ill patients in the intensive care unit: a systematic review

**DOI:** 10.1590/S1679-45082014RW2955

**Published:** 2014

**Authors:** Lucas Lima Ferreira, Luiz Carlos Marques Vanderlei, Vitor Engrácia Valenti

**Affiliations:** 1 Universidade Estadual Paulista “Júlio de Mesquita Filho”, Presidente Prudente, SP, Brazil.

**Keywords:** Physical therapy modalities, Electric stimulation, Intensive care units

## Abstract

**Objective:**

To analyze the outcomes enabled by the neuromuscular electric stimulation in critically ill patients in intensive care unit assisted.

**Methods:**

A systematic review of the literature by means of clinical trials published between 2002 and 2012 in the databases LILACS, SciELO, MEDLINE and PEDro using the descriptors “intensive care unit”, “physical therapy”, “physiotherapy”, “electric stimulation” and “randomized controlled trials”.

**Results:**

We included four trials. The sample size varied between 8 to 33 individuals of both genders, with ages ranging between 52 and 79 years, undergoing invasive mechanical ventilation. Of the articles analyzed, three showed significant benefits of neuromuscular electrical stimulation in critically ill patients, such as improvement in peripheral muscle strength, exercise capacity, functionality, or loss of thickness of the muscle layer.

**Conclusion:**

The application of neuromuscular electrical stimulation promotes a beneficial response in critically patients in intensive care.

## INTRODUCTION

Currently, advances in care for Intensive Care Unit (ICU) patients have improved results and survival rates for this population of patients.^(1, 2)^ As more patients survive the acute disease, long-term complications become more apparent, some likely leading to greater deficiency, with prolonged stays and rehabilitation under intensive care.^(3)-8)^

Muscular weakness in critically ill patients is one of the most common problems in ICU patients,^(9, 10)^ it is diffuse and symmetric, affecting striated appendicular and axial skeletal muscles.^(9, 11)^ Within this context, early physical and occupational treatment in these individuals has been showing rapid growth, although pertinent literature is still scarce.^(12, 13)^ The intensive care physical therapist treats this dysfunction by means of techniques such as early mobilization and neuromuscular electrical stimulation (NMES), among others.^(11)^

According to the American Physical Therapy Association (APTA), NMES is the application of therapeutic electrical stimuli applied to muscle tissue through a sound peripheral nervous system in order to restore motor and sensory functions.^(14)^ Muscle contraction induced by electrical activation occurs differently from physiologically induced muscle contraction.^(15)^

In voluntary contraction, the recruitment order comes in accordance with Henneman’s principle, that is, slow motor units (type I) are used for small efforts, while rapid motor units (type II) are gradually recruited when there are greater levels of strength production.^(15)^ During NMES, recruitment occurs inversely: the rapid fibers are the first to be recruited, and this phenomenon happens because the electrical stimuli is applied externally to the nerve endings and because the larger cells, with low axonal input, are more excitable.^(14, 15)^

However, a search conducted in specialized databases did not indicate systematic literature reviews of meta-analyses that confirm benefits or harm afforded by NMES for the critically ill patient in an intensive care environment. Thus, the present study had the objective of performing a systematic review of literature in order to clarify the outcomes caused by NMES application in critically ill patients in the ICU.

RETRACTED

## METHODS

This was a systematic review of literature, based on the PRISMA guideline.^(16)^

### Eligibility criteria and source selection

The search for articles involving intended clinical outcomes was made in the Latin-American and Caribbean Literature (LILACS), Scientific Electronic Library Online (SciELO), Medical Literature Analysis and Retrieval System Online (MedLine/PubMed), and Physiotherapy Evidence Database (PEDro) databases. The articles were obtained by means of the following key words: “intensive care unit”, “physical therapy”, “physiotherapy”, “electrical stimulation”, and “randomized controlled trials” with the Boolean descriptor “and”.

The search for references was limited to articles written in Portuguese, English, or Spanish, published between 2002 and 2012.

### Inclusion and exclusion criteria

At the end of the analysis, only the clinical trials that covered the performance of some modality of NMES in gravely ill adult ICU patients were included.

Letters, summaries, dissertations, theses, and case reports were excluded, as well as studies that used children or animal models.

### Data analysis

Qualitative analysis of the studies identified was made with the presentation of data in the form of tables, with description of the following characteristics: author, sample characteristics, intervention, primary variables of the outcomes, and significant results.

## RESULTS

Forty-three relevant studies were identified, 39 of which were excluded for not having the methodological outlining stipulated in the present study (Figure 1). Thus, four clinical assays were included ^(17)-20)^ that addressed the criteria established for the intended outcome.

RETRACTED

**Figure 1:** Flowchart of the article selection strategy

The information on the studies included is summarized on Chart 1. Among the studies selected, three used a control group for comparison of results.^(17)-19)^ Sample size varied from 8 to 33 subjects, of both genders, with a mean age of 52 to 79 years, submitted to invasive mechanical ventilation (IMV).

Table 1 shows the characteristics of NMES used in the clinical trials. These characteristics diverged as to modulation of the device and time of application of the technique, as one was late,^(17)^ two were early,^(18, 20)^ and one associated early and late NMES.^(19)^

**Chart 1:** Characteristics of the selected randomized clinical trials focusing on neuromuscular electrical stimulation (NMES) in the critically ill patient

Author	Sample characteristics	Intervention	Primary outcome variables	Significant results
Zanotti et al.^(17)^	n=24 (GE: 12; CG: 12)	EG: active exercises and NMES in LLs (30 minutes)	PMS and days necessary for transfer from bed to chair	Increase in PMS in both groups, more expressive in the EG; the EG was able to transfer from bed to chair in fewer days
	chronic COPD, undergoing IMV, bed-ridden for more than 30 days, with severe peripheral atrophy			
		CG: only active exercises;		
		Time: 5 times a week during 4 weeks		
Gerovasili et al.^(18)^	n=26 (EG: 13; CG: 13)	EG: daily sessions of NMES in LLs (55 minutes)	Muscle diameter by ultrasonography	Decrease in muscle diameter of femoral quadriceps in both groups, with smaller reduction in the EG
	ICU patients, undergoing IMV, with APACHE II ≥ 13			
		CG: not specified		
		Time: from 2^nd^ to 9^th^ day in ICU		
Gruther et al.^(19)^	n=33 (EG: 16; CG: 17)	EG: early NMES (30-60 minutes) with time of hospital stay >1 week; and late with hospital stay <2 weeks;	Muscle diameter of the femoral quadriceps by ultrasonography	Thickness of the muscle layer decreased in both groups of early NMES. In the late NMES group, there was an increase in muscle mass
	ICU patients, stratified into 2 groups: early and late			
		CG: placebo		
		Time: 5 times a week for 4 weeks		
Poulsen et al.^(20)^	n=8 Patients admitted to the ICU with septic shock, undergoing IMV	Unilateral NMES (60 min) with contralateral thigh as paired control associated with conventional physical therapy Time: 7 consecutive days	Assessment of muscle mass by computed tomography of the thigh	There was no difference between baseline and post-NMES values in muscle volume between the stimulated and non-stimulated sides
		Tempo: 7 dias consecutivos		

EG: experimental group; CG: control group; COPD: chronic obstructive pulmonary disease; IMV: invasive mechanical ventilation; LLs: lower limbs; PMS: peripheral muscle strength; ICU: intensive care unit; APACHE II: Acute Physiology and Health Evaluation II.

RETRACTED

Of the four studies included in this review, three showed significant benefits of NMES application in gravely ill ICU patients,^(17)-19)^ such as improvement in peripheral muscle strength, exercise capacity, functionality or thickness of muscle layer loss.

## DISCUSSION

The present review detected a beneficial response for the applications of NMES modalities in severely ill ICU patients. It also determined that studies performed at a late phase with more chronic and debilitated patients, and which focused on the increase of muscle mass, had more satisfactory results.^(17, 19)^

The studies included in this review demonstrated that the performance of NMES in the gravely ill patient represents a safe, viable, and well tolerated intervention.^(17)-20)^ Serious adverse reactions were uncommon, with no need to interrupt therapy – interruption is normally associated with asynchrony between the patient and the mechanical ventilator.

Zanotti et al.^(17)^ compared a protocol of active appendicular exercises to NMES in patients with severe chronic obstructive pulmonary disease who were bed-ridden and under prolonged IMV. The NMES protocol consisted of the application of biphasic square pulse wave with surface electrodes on the quadriceps and gluteus muscles bilaterally, in 30-minutes sessions, five times a week, for 4 weeks. Each session began with a frequency of 8Hz and 25 microseconds (ms) pulse width during five minutes, and then 35Hz frequency with a 35ms pulse width for 25 minutes. The authors noted that the group that received NMES obtained a significantly greater increase in muscle strength when compared to participants of the exercise group.

Another study^(18)^ with gravely ill patients applied NMES concomitantly to the quadriceps and fibularis longus from the second to the ninth day of hospitalization. The protocol consisted of daily sessions with 45Hz frequency and pulse width of 40ms during 55 minutes. The group submitted to the intervention progressed with a smaller muscle mass in comparison with the control group.

Gruther et al.^(19)^ applied NMES to the quadriceps of 17 gravely ill patients using a protocol composed of 50Hz frequency, 35ms pulse width, for 30 to 60 minutes, during four weeks. These authors observed a delay in decrease of the mean thickness of the muscle layer in patients submitted to NMES as of the second week of ICU stay.

A recent study^(20)^ analyzed the addition of NMES to the treatment of eight patients with septic shock undergoing IMV in the ICU. The protocol was composed of seven sessions, with 60 minutes duration each, in which NMES was applied with a frequency of 35Hz and pulse width of 30ms to the quadriceps unilaterally, using the contralateral quadriceps as control. No significant difference was noted in the muscle volume between the stimulated and non-stimulated sides. The authors attribute the fact to the intensity of the current used and to the underlying pathology of the patients that occurred with systemic manifestations.

RETRACTED

In general, the four studies^(17)-20)^ included in the present review adopted NMES protocols that varied in frequency from 35 to 50Hz and pulse width of 30 to 40ms, with an intensity that provoked visible contraction, in sessions that lasted between 30 and 60 minutes, during 1 to 4 weeks. Such variations in the protocols analyzed hinder the comparison and postulation of plausible evidence for clinical practice of the said resource.

It is important to point out that the patients studied were submitted to IMV, and neuromuscular abnormalities acquired in the ICU are common in this population, since prolonged IMV is considered a risk factor for the development of serious muscle weakness, besides promoting damage to functional performance, with a strong correlation between the time free from IMV and the functional performance of the patient.^(21)^ One prospective cohort study carried out in four hospitals detected severe muscle weakness in 25% of the gravely ill patients submitted to IMV for more than 1 week.^(5)^

The affirmation that better results were obtained with the late application of NMES was verified through analysis of the study by Gruther et al.,^(19)^ which evaluated the effects in two groups of patients: (1) early, intended to prevent loss of muscle mass; (2) late, with the objective of reversing muscle hypotrophy. Both groups were divided into subgroups of intervention and control. A significant decrease was shown in the thickness of the muscle layer of the group that received early intervention (in both subgroups), demonstrating that NMES did not prevent muscle mass loss. On the other hand, in the group that received late electrostimulation, the intervention group showed a significant increase in muscle mass when compared to the control subjects.

One plausible explanation for NMES not having affected muscle mass loss when applied early to severely ill patients is the fact that immobilization, even when during a short period of time, promotes a catabolic state in the muscle, resulting in significant loss of muscle mass and decrease in strength, and is more accentuated during the first three weeks of hospital stay.^(22)^

In two trials analyzed,^(19, 20)^ NMES was applied to the quadriceps muscle due to the accentuated loss of mass that occurred in this muscle group during the first weeks of ICU stay. However, it was noted that such a loss was not affected by the daily application of NMES, and this may have happened as a results of the possible correlation between NMES and the severity of the underlying pathology which may have affected the excitability of the muscle tissue.^(20)^

This study had as limitations the reduced number of randomized clinical trials with adequate methodological assessment, the reduced sample size of the studies analyzed, variation of the parameters used for electrostimulation, and the different times of application and use of the interventions, as well as the heterogeneity of the outcomes evaluated, which compromise the comparisons of the effects found among the authors.

RETRACTED

Finally, it is important to consider that the diversity of NMES protocols found and of the methods of evaluation limit the direct comparison among the groups. There is no consensus as to adequate modulation, so as to promote strong contractions with a minimum of muscle fatigue. Nevertheless, the evidence currently available on the effects of NMES on the gravely ill patient is limited, due to the scarcity of studies published on the theme.

## CONCLUSION

The application of electrostimulation promotes a beneficial response characterized by improved peripheral muscle strength, exercise capacity, functionality, or thickness of muscle layer loss, in gravely ill patients in an intensive care unit. The most satisfactory results were obtained when neuromuscular electrical stimulation was applied later. In terms of practical application, neuromuscular electrical stimulation is viable and easily inserted into the intensive care environment, helping to correct peripheral neuropathies and to decrease time of stay of patients in the intensive care unit.

**Table 1:** Characteristics of neuromuscular electrical stimulation (NMES) in the clinical trials analyzed

NMES modulation	Zanotti et al.^(17)^	Gerovasili et al.^(18)^	Gruther et al.^(19)^	Poulsen et al.^(20)^
Frequency (Hz)	35	45	50	35
Pulse width (ms)	0.35	0.40	0.35	0.30
Intensity	Non-stimulated	Visible contraction	Visible contraction	Visible contraction
Time of session (minutes)	30	55	30 a 60	60
Stimulated muscle group	Quadriceps e gluteus	Quadriceps and fibularis longus	Quadriceps	Quadriceps
